The article "Effect of HCH Nutrition Management Combined with Early Exercise Nursing on Nutrition Status and Postoperative Rehabilitation of Patients after Gastric Cancer Surgery" was retracted in 2023. Reasons: signs of a paper mill; suspected computer-generated content; unreliable results or conclusions; lack of ethics approval or compliance.

# Effect of HCH Nutrition Management Combined with Early Exercise Nursing on Nutrition Status and Postoperative Rehabilitation of Patients after Gastric Cancer Surgery

**DOI:** 10.1155/2022/2813050

**Published:** 2022-08-18

**Authors:** Zengfen Pang, Yuanyuan Li, Amei Huang, Xianghong Li, Yuping Liu, Yingtao Meng

**Affiliations:** Shandong Cancer Hospital and Institute, Jinan, China

## Abstract

**Objective:**

The study aimed to analyze the effect of hospital-community-family (HCH) nutrition management combined with early exercise nursing on nutrition status and postoperative rehabilitation of patients after gastric cancer surgery.

**Methods:**

A total of 80 patients with gastric cancer admitted from January 2019 to June 2021 were selected and divided by the odd-even grouping method into two groups, i.e., 40 cases in the control group adopting routine nursing combined with early exercise nursing and 40 cases in the study group adopting HCH nutrition management; the nutrition status and postoperative rehabilitation of the two groups were compared.

**Results:**

The times of feeding, bowel sound, anal exhaust, and defecation in the study group after surgery were shorter than those in the control group, with a difference of statistical significance (*P* < 0.05). 3 months after discharge, the scores of Patient-Generated Subjective Global Assessment (PG-SAG) in the study group were lower than those in the control group, while the body mass index (BMI), prealbumin, albumin, hemoglobin, and the score of the Gastrointestinal Quality of Life Index (GIQLI) were higher than those of the control group (*P* < 0.05).

**Conclusion:**

Hospital-community-family nutrition management combined with early exercise nursing can improve the postoperative nutrition status of patients undergoing gastric cancer surgery and advance the time of postoperative exhaust and defecation.

## 1. Introduction

As a common tumor of the digestive system, gastric cancer ranks second in morbidity and mortality among all malignant tumors in China. Malnutrition is common in patients with gastric cancer due to the tumor itself and gastrectomy [1]. According to incomplete statistics, 48% of newly diagnosed tumor patients suffer from severe malnutrition, and 17% suffer from mild to moderate malnutrition [2]. However, early exercise after gastric cancer surgery can facilitate tissue regeneration and repair in patients, promote intestinal function rehabilitation, and reduce adverse reactions caused by long-term bed rest [3]. Therefore, the implementation of early exercise for patients aims to improve compliance with early exercise after surgery and promote rehabilitation. Meanwhile, postoperative malnutrition will increase medical expenses and economic burden; thus, necessary nutritional support can provide necessary nutrients for disease rehabilitation, prevent complications, and improve the clinical outcome of patients. First proposed by the Cancer Nutrition and Support Treatment Committee of the China Anti-Cancer Association, hospital-community-family (HCH) nutrition management is a nutrition management mode with the characteristics of hierarchical management, three-level linkage, seamless connection, and two-way circulation, which extends nutrition management from hospitals to communities and families and expands nutritional objects to patients and their family members, so as to improve the nutrition management level [4]. This experiment is designed to improve the rehabilitation level of postoperative patients with gastric cancer, which adopts HCH nutrition management combined with early exercise nursing to analyze the rehabilitation effect of patients. It is reported as follows.

## 2. Data and Methods

### 2.1. Clinical Data

A total of 80 patients with gastric cancer admitted from January 2019 to June 2021 were selected and divided by the odd-even grouping method into two groups. There were 40 patients in the control group (male: 21, female: 19), with an age ranging from 45 to 72 (58.84 ± 5.28) years; histological classification: 25 cases of low-differentiated adenocarcinoma, 10 cases of high-differentiated adenocarcinoma, and 5 cases of medium-low differentiated adenocarcinoma; tumor stage: 10 cases in stage I, 18 cases in stage II, and 12 cases in stage III; 11 cases of radical total gastrectomy and 29 cases of radical subtotal gastrectomy. There were 40 cases in the study group (male: 23, female: 17), with an age ranging from 45 to 72 (59.25 ± 5.31) years; histological classification: 23 cases of low-differentiated adenocarcinoma, 12 cases of high-differentiated adenocarcinoma, and 5 cases of medium-low differentiated adenocarcinoma; tumor stage: 8 cases in stage I, 20 cases in stage II, and 12 cases in stage III; 14 cases of radical total gastrectomy and 26 cases of radical subtotal gastrectomy. The baseline data of the two groups were homogeneous (*P* > 0.05), indicating comparability.

Inclusion criteria were as follows: (1) patients enrolled conform to the criteria of gastric cancer through a comprehensive examination of clinical manifestations, imaging, and pathology [5]; (2) patients voluntarily undergo gastric cancer surgery; (3) with normal liver and kidney function; (4) the baseline data of patients are complete; (5) patients and their families are informed of the research and sign the consent form.

Exclusion criteria were as follows: (1) patients with blood diseases, immunodeficiency diseases, and severe infections; (2) patients with schizophrenia and cognitive abnormalities; (3) recent functional gastrointestinal disorders; (4) patients with rerecurrence of gastrointestinal tumors; (5) patients with severe malnutrition before surgery.

### 2.2. Methods

The control group was treated with routine nursing combined with early exercise nursing, which explains the basic procedures of gastric cancer surgery and postoperative precautions through a rehabilitation guide and video presentation before surgery and implements enteral and parenteral nutrition according to the doctor's advice after surgery. The postoperative changes of the disease were closely monitored in order to effectively prevent complications. When discharged from the hospital, a diet manual was issued, requiring the patient to eat accurately and take early exercise after surgery. (1) Extremely early exercise (6∼24 h after surgery). After surgery, the patient rests in a supine position with sandbags placed on the abdomen for about 6 hours, and the patient was assisted to change his posture after waking up. After 12 h, the patient took a semisupine position and turned over, with one hand covering his abdomen and turning slowly with the other hand on the edge of the bed. The patient was instructed to breathe with abdominal muscles, inhale and exhale at a uniform depth, and alternately do abdominal breathing and chest breathing and instructed to contract the anus for 30 minutes each time, 1∼2 times per day. (2) Sub-early exercise (25∼48h after surgery). Patients were instructed to do upper limb activities, including fist clenching, elbow joint flexing and stretching, arm lifting, and shoulder rotating and lower limb activities: knee joint flexing and stretching, hip joint abduction, straight leg raising, and alternate cycling activities. (3) Early exercise (>48 h after surgery). Except for patients with contraindications, patients were encouraged to walk beside the bed on the first day after surgery or to sit up, stand up, walk with the support of the bed after 48 hours, and gradually walk outside the ward. The distance of the first walk after surgery was 25∼50 m and gradually increased to 50∼100 m when discharged from the hospital. Patients were encouraged to independently complete daily activities such as eating and washing and to massage the abdomen clockwise about 300 times after surgery, with one hand protecting the incision, and it was best to produce a mild heat sensation in the abdomen. The study group adopted the HCH nutrition management based on the control group. (1) Establishment of an HCH nutrition management team. The team consisted of 1 clinical dietitian, 2 clinicians, 2 primary nurses, 4 community nurses, and family members of the patient. Except for family members of the patient, the rest of the team received nutrition knowledge training and participated in this nursing intervention only after passing the training and examination. (2) Establishment of nutrition archives. When the patient was discharged from the hospital, the dietitian evaluated the nutrition status of the patient, worked out a nutrition plan together with the doctor in charge, and taught the patient and his family about nutrition knowledge and nutrition prescriptions through health guides, short videos, pictures, and texts, etc. The community nurse regularly tracked the nutrition intake of the patient, evaluated the nutrition risks and indicators, and gave feedback to the dietitian. The family members supervised the diet of the patient and kept a diet diary. (3) Practice content. Before discharge, patients followed the WeChat group and WeChat official account for the regular push of nutrition and health knowledge, providing health consultation and nutrition guidance for patients and their families. The hospital mainly carried out the three-level nutrition diagnosis for patients and implemented precise nutrition therapy; the community mainly provided nutrition consultation and education for patients and their families, regularly screened nutrition status, and implemented individualized and targeted nutrition intervention. The family primarily encouraged the patients to develop good and healthy living habits, as well as to actively record the nutrition levels and risks; they also encouraged patients to participate in sports activities and to take oral nutrition supplements. Patients were required to keep records of their daily diet, including daily food intake, food type, urination, and defecation and record weekly weight changes. In case of decreased food intake, continuous diet decline, involuntary weight loss, etc., patients should contact the community nurse immediately and communicate with the dietitian in time. The intervention lasted for 3 months.

### 2.3. Observation Indexes

(1) We compare the starting time of postoperative feeding, bowel sound, anal exhaust, and anal defecation between the two groups. (2) We compare the nutritional risk at discharge and 3 months after discharge between the two groups and adopt PG-SAG [6] for assessment: good nutrition: Grade A (0∼1); suspected or mild malnutrition: Grade B (2∼3); moderate malnutrition: Grade C (4∼8); severe malnutrition: Grade D (>8). (3) We compare the BMI, prealbumin, albumin, and hemoglobin at discharge and 3 months after discharge between the two groups. (4) We compare the quality of life at discharge and at 3 months between the two groups and adopt the Gastrointestinal Quality of Life Index (GIQLI) [7], which has 36 items and each item scores 4∼0 points from zero to severe. The higher the total score, the better the quality of life.

### 2.4. Statistical Method

With SPSS20.0 statistical software, the measurement data were expressed by (±*s*) and verified by the *T* test. The count data were expressed in (%) and verified by ^2^ tests, which indicated statistical difference (*P* < 0.05).

## 3. Results

### 3.1. Comparison of Postoperative Rehabilitation Progress between the Two Groups

The starting times of the postoperative feeding, bowel sound, anal exhaust, and anal defecation in the study group were shorter than those in the control group, with statistical significance (*P* < 0.05) as shown in Table 1.

### 3.2. Comparison of Nutritional Risks between Two Groups at Discharge and 3 months after Discharge

The PG-SAG score between the two groups at discharge was compared (*P* > 0.05). The PG-SAG scores of the two groups 3 months after discharge were lower than those at discharge (*P* < 0.05), and the PG-SAG score of the study group was lower than that of the control group (*P* < 0.05), as shown in Table 2.

### 3.3. Comparison of Anthropometric Measurements of the Two Groups at Discharge and 3 months after Discharge

The BMI, prealbumin, albumin, and hemoglobin between the two groups at discharge were compared (*P* > 0.05). The BMI, prealbumin, albumin, and hemoglobin of the two groups 3 months after discharge were higher than those at discharge (*P* < 0.05), which showed the anthropometric measurements of the study group were higher than those of the control group (*P* < 0.05), as shown in Table 3.

### 3.4. Comparison of the GIQLI Score of Life Quality at Discharge and 3 months after Discharge between the Two Groups

The life quality score of the two groups at discharge was compared (*P* > 0.05). The life quality score of the two groups 3 months after discharge was higher than that at discharge (*P* < 0.05), which showed the life quality score of the study group was higher than that of the control group (*P* < 0.05), as shown in Table 4.

## 4. Discussion

As the main method for the treatment of gastric cancer, surgery causes delayed rehabilitation of gastrointestinal function due to major trauma, strong invasion and stimulation of intraoperative anesthesia, and traction, which directly affects the feeding and rehabilitation progress of the patients after surgery. A number of practices have proved that early exercise can promote the rehabilitation of gastrointestinal function after surgery, reduce the occurrence of postoperative complications, and enable patients to return to normal life as soon as possible [8, 9]. Therefore, early exercise should be adopted by patients undergoing gastric cancer surgery and divided into super-early exercise, sub-early exercise, and early exercise, including posture change, breathing exercise, turning over, limb movement, off-bed activities, and daily activities, which can correspondingly improve the autonomic nerve function that controls visceral activities, reduce the excitability of the sympathetic nerve, and increase the tension of the vagus nerve. In addition, it can promote abdominal blood circulation, increase the intra-abdominal blood flow, and provide adequate blood perfusion and oxygen supply to the gastrointestinal tract [10]. Furthermore, early exercise can promote gastrointestinal peristalsis and friction between intestinal loops, and reduce the resistance between the gastrointestinal tract and peritoneum, mesentery, and other tissues, so as to maintain stable visceral activities, reduce gastrointestinal discomfort, and facilitate postoperative rehabilitation of patients as soon as possible after surgery. Meanwhile, malnutrition is a common complication of cancer patients, with an incidence of up to 67%, especially in gastrointestinal tumor patients, with a higher incidence of malnutrition [11]. Nutrition management is an important method for maintaining the tumor patient's nutrition status. However, due to insufficient awareness of nutrition and shortage of medical resources, the nutrition status of most patients has not been corrected at discharge, and the nutrition supply is insufficient after discharge, which is inclined to increase the degree of malnutrition. HCH nutrition management is a new mode of nutrition management in recent years, which can give full play to the management strength and effect of hospital, community, and family, extend the content, broaden the scope, and increase the objects of nutrition management, thus improving the level of nutrition management [12].

In this study, the starting time of postoperative feeding, bowel sound, anal exhaust, and anal defecation in the study group was shorter than those in the control group, with statistical significance (*P* < 0.05). The results have shown that HCH nutrition management combined with early exercise nursing can promote gastrointestinal peristalsis of patients with gastric cancer after surgery, facilitate refeeding as soon as possible, and further improve the postoperative functions of patients. The reason is that early exercise nursing with instructed activities step by step can increase abdominal blood flow, improve gastrointestinal peristalsis, and maintain stable visceral activities, thus speeding up postoperative rehabilitation of patients. Furthermore, it can provide professional nutrition management for patients, give full play to the core role of nutrition management in the hospital, and maintain the stability of the internal environment and vital signs of the patients; it focuses on maintaining and improving the organ functions of patients and provides precise nutrition therapy, in order to provide patients with necessary nutrition support and promote their rehabilitation after surgery as soon as possible.

In this study, the PG-SAG score of the study group was lower than that of the control group 3 months after discharge, while the BMI index, prealbumin, albumin, and hemoglobin were higher than those of the control group, and the GIQLI score of quality of life was higher than that of the control group (*P* < 0.05). The results have shown that HCH nutrition management combined with early exercise nursing can improve the nutrition status and quality of life of patients with gastric cancer after discharge. Analysis of reasons: In contrast to ordinary patients, gastric cancer patients suffer from stomach function loss and tumor cell invasion to multiple organ functions, and most of them are malnourished. The HCH nutrition management is adopted to provide patients with a three-level nutrition diagnosis and precise nutrition treatment in the hospital to improve their nutrition level. However, there are still some patients with poor recovery of nutrition status, coupled with the shortage of medical resources and economic burden, which results in insufficient nutrition supply and demand for patients and aggravated malnutrition after discharge. Therefore, exerting full play to the role of community nutrition management and the supervision and management of patients and their families, providing regular and professional nutrition supply for patients, and giving full play to the cooperation between doctors and patients can improve the nutrition management ability of patients. Meanwhile, with the help of Internet platforms such as WeChat group and WeChat official account, it can realize barrier-free communication between doctors and patients and timely information feedback, solve the problems encountered by patients after discharge, make patients develop good and healthy living habits, and improve their nutrition status. In addition, family is the basic unit of nutrition management and an important place to realize individual nutrition management. Family members play a supervisory role in requiring the patients to record their weight, food intake, urination, and defecation every week. Oral nutritional supplements can also effectively prevent malnutrition, promote rehabilitation, and improve the nutrition status of patients.

In conclusion, hospital-community-family nutrition management combined with early exercise nursing will improve the nutrition status of patients with gastric cancer surgery after discharge, shorten the time of postoperative exhaust and defecation, and improve their quality of life, thus establishing a good rehabilitation management model for patients, which is of high clinical significance and worthy of further clinical exploration.

## Figures and Tables

**Table 1:** Comparison of postoperative rehabilitation progress between the two groups (h).

Group	Number of cases	Starting time of postoperative feeding	Bowel sound	Anal exhaust	Anal defecation
Study group	40	38.54 ± 5.28	15.24 ± 3.15	44.25 ± 8.46	42.54 ± 3.51
Control group	40	49.24 ± 5.34	21.89 ± 4.28	56.51 ± 8.52	51.95 ± 4.27
*T*		9.012	7.914	6.458	10.767
*P*		<0.001	<0.001	<0.001	<0.001

**Table 2:** Comparison of PG-SAG scores of nutritional risks at discharge and 3 months after discharge between the two groups (score).

Group	Number of cases	At discharge	3 months after discharge	*t*	*P*
Study group	40	4.05 ± 0.52	1.15 ± 0.21	32.705	<0.001
Control group	40	3.99 ± 0.51	2.53 ± 0.35	14.928	<0.001
*T*		0.521	21.383		
*P*		0.604	<0.001		

**Table 3:** Comparison of anthropometric measurements of the two groups at discharge and 3 months after discharge.

Group	BMI (kg/m2)		Albumin (g/L)		Prealbumin (g/L)		Hemoglobin (g/L)	
	At discharge	3 months after discharge	At discharge	3 months after discharge	At discharge	3 months after discharge	At discharge	3 months after discharge
Study group (*n* = 40)	18.95 ± 1.24	22.18 ± 0.96^a^	29.89 ± 2.15	36.52 ± 2.42^a^	168.85 ± 18.46	245.25 ± 19.10^a^	109.85 ± 5.46	128.53 ± 3.46^a^
Control group (*n* = 40)	19.10 ± 1.31	21.27 ± 0.82^a^	30.16 ± 2.21	33.84 ± 2.51^a^	170.12 ± 19.20	218.24 ± 18.65^a^	110.12 ± 5.51	121.05 ± 3.19^a^
*T*	0.526	4.559	0.554	4.861	0.302	6.399	0.220	10.052
*P*	0.600	<0.001	0.581	<0.001	0.764	<0.001	0.826	<0.001

*Note.* ^a^ *P* < 0.05, compared with that at discharge.

**Table 4:** Comparison of the GIQLI score of life quality at discharge and 3 months after discharge between the two groups (score).

Group	Number of cases	At discharge	3 months after discharge	*t*	*P*
Study group	40	89.85 ± 8.51	128.12 ± 5.46	23.938	<0.001
Control group	40	90.12 ± 8.74	112.05 ± 5.38	13.514	<0.001
*T*		0.140	13.259		
*P*		0.889	<0.001		

## Data Availability

The simulation experiment data used to support the findings of this study are available from the corresponding author upon request.
